The article "Breast MRI Segmentation and Ki-67 High- and Low-Expression Prediction Algorithm Based on Deep Learning" was published in 2022. Journal: Comput Math Methods Med.

# Breast MRI Segmentation and Ki-67 High- and Low-Expression Prediction Algorithm Based on Deep Learning

**DOI:** 10.1155/2022/1770531

**Published:** 2022-10-04

**Authors:** Yuan-Zhe Li, Yin-Hui Huang, Xian-yan Su, Zhen-qi Gu, Qing-Quan Lai, Jing Huang, Shu-Ting Li, Yi Wang

**Affiliations:** ^1^Department of CT/MRI, The Second Affiliated Hospital of Fujian Medical University, Quanzhou 362000, China; ^2^Department of Neurology, Jinjiang Municipal Hospital, Quanzhou 362000, China; ^3^Galactophore Department, The First School of Clinical Medicine, Zhejiang Chinese Medical University, 548 Binwen Road, Hangzhou 310000, China

## Abstract

**Results:**

The DSC, PPV, and sensitivity of our combined model are 0.94, 0.93, and 0.94, respectively, with better segmentation performance. And we compare with the segmentation frameworks of other papers and find that our combined model can make accurate segmentation of breast tumors.

**Conclusion:**

Our method can adapt to the variability of breast tumors and segment breast tumors accurately and efficiently. In the future, it can be widely used in clinical practice, so as to help the clinic better formulate a reasonable diagnosis and treatment plan for breast cancer patients.

## 1. Introduction

Tumors are the leading cause of death worldwide. Breast cancer is the malignant tumor with the highest incidence of female malignancies, and its incidence is increasing year by year and younger women are being diagnosed with it [1, 2]. Breast cancer is a very heterogeneous illness that can be categorized into four molecular types: luminal A, luminal B, HER-2, and basal-like, according to the rapid progress of tumor molecular biology research. The disease manifestation, responsiveness to treatment, and other clinical behaviors of breast cancer patients with distinct molecular types varied significantly [3–6]. The Ki-67 protein is a nuclear antigen linked to cell proliferation that can accurately reflect the proliferative activity of malignant tumors, making it a useful indicator of tumor aggressiveness [7–9]. Recent studies have found that the proliferation marker Ki-67 provides important prognostic information and may contribute to the evaluation and improvement of treatment in prognostic ER-positive breast cancer [10]. Although some relapse, around 70% of human breast cancer tumors are ER-positive and have a favorable prognosis.

The Ki-67 index, a proliferation marker, has been utilized to distinguish luminal B from luminal A tumors in estrogen receptor-positive individuals and is a consistent sign of more aggressive breast cancer growth [11]. Patients with the luminal B subtype had a higher rate of proliferation and a worse prognosis than those with the luminal A subtype. Luminal B tumors have reduced estrogen-related gene expression and a higher Ki-67 index, making them a subgroup of ER-positive patients with a poor prognosis who may benefit from adjuvant treatment. It is critical to recognize groups [12–14]. Individuals with lower Ki-67 levels have a basic pathological complete response (PCR) after treatment, whereas patients with high Ki-67 expression are considered a high-risk category in terms of prognosis, according to new research [15]. The Ki-67 expression determination rule is follows: the proportion of positive cancer cells in the sample is counted, and the proportion greater than 14% is defined as high expression; otherwise, it is low expression [16]. Data mining of the Ki-67 high and low expression based on advanced algorithms [17–19] may assist in the prediction. If a reliable prediction method for breast cancer patients to avoid invasive damage can be found to predict Ki-67 before pathological examination, it will be very beneficial for doctors to formulate later treatment plans and provide more useful treatment options basis.

The article "Breast MRI Segmentation and Ki-67 High- and Low-Expression Prediction Algorithm Based on Deep Learning" was published in 2022. Journal: Comput Math Methods Med.

With the improvement, development, and application of various MRI techniques, because of its unique imaging characteristics and advantages, it has become an important supplementary method after mammography and ultrasonography [20]. MRI has a strong ability to distinguish between different soft tissue structures, especially for various breast lesions [21]. Some studies have shown that its diagnostic sensitivity for breast cancer reaches 94%-99%, and MRI also has higher accuracy and objectivity for the localization of breast lesions [22]. At the same time, it can be observed whether the lesion has various effects on the surrounding tissues, such as whether the lesion involves adjacent muscle groups such as the pectoralis major, whether it invades or destroys the adjacent bone structure, and whether there is abnormal signal changes such as edema in the surrounding normal soft tissue [23]. Especially when a suspicious breast cancer is found, it is more valuable to assess whether there is metastasis in the lymphatic drainage areas of the breast, such as the axilla, subclavian, and posterior sternum, which is helpful for the clinical staging of breast cancer and assists early clinical development. Patients' prognoses and survival times can be improved by using the appropriate treatment options [24].

A technique that is noninvasive and nonharmful. Diffusion weighted imaging (DWI) is a development of magnetic resonance imaging (MRI) technology that has been widely employed in breast imaging tests. It can detect the diffusion movement of water molecules in human tissues. Information such as direction and degree of restriction indirectly reflect changes in tissue microstructure [25, 26]. The apparent diffusion coefficient (ADC) is a quantitative metric that closely represents biological tumor properties such as vascular anatomy and water content [27]. Imaging analysis of breast tumor heterogeneity based on diffusion weighted imaging is currently attracting great attention internationally. Previous studies have found some significant DWI imaging features of breast molecular typing and the relationship between ADC values in tumors and surrounding stromal regions and pathological status [24, 28], but ADC values in tumors and surrounding stromal regions were found. The heterogeneous signaling patterns and the use of these features to predict molecular typing have not been studied.

The article "Breast MRI Segmentation and Ki-67 High- and Low-Expression Prediction Algorithm Based on Deep Learning" was published in 2022. Journal: Comput Math Methods Med.

Today, deep learning methods are applied to many pattern recognition tasks with good results, in which convolutional neural network algorithms can automatically learn image features [29]. Among them, Piantadosi et al. [30] accurately segmented the breast by applying CNN on 3D MRI. They also used an appropriate projection fusion method to merge U-Net with CNN for multiplanarity, allowing for multiprotocol applications. The U-Net neural network was appropriately modified by Piantadosi et al. [31]. The network enables accurate segmentation of 3D breast MRI. Zhang et al. [32] used the U-Net framework incorporating a fully convolutional residual neural network for accurate segmentation of breast MRI. It has the potential to provide a reliable and efficient approach for processing huge volumes of MRI data and quantitative breast density analysis. To accurately segment breast MRI and catch mistakes, Kakileti et al. [33] suggested a cascaded CNN architecture. The suggested system can automatically detect breast regions regardless of picture capture or angle, allowing for image and video analysis.

This paper proposes a tumor segmentation and prediction framework based on the combination of improved attention U-Net and SVM. The framework first improves on attention U-Net by introducing coefficients for learning multidimensional attention. It causes the attention mechanism in the segmentation process to devote more attention to the main situation. At the same time, the segmented breast MRI results and corresponding labels were input into the SVM classifier to accurately predict the expression of Ki-67.

## 2. Materials and Methods

### 2.1. Construction of the Dataset

#### 2.1.1. Data Acquisition

We collected breast MRI data from 164 patients from the Second Affiliated Hospital of Fujian Medical University. According to the pathology report, there were 98 cases with high expression of Ki-67 (greater than or equal to 14%) and 66 cases with low expression of Ki-67 (less than 14%). Inclusion criteria are as follows: (1) have had breast MRI examination before surgery and (2) postoperative pathology report accurately indicated the molecular subtype of breast cancer with Ki-67 classification. Patients were scanned in the prone position using a 3.0 T MRI scanner (PHILIPS, Ingenia 3.0 T) with a dedicated phased array 8-channel breast coil. The identical imaging strategy was used on all of the patients. The breast DWI technique included a DWI sequence (TR/TE = 6000 ms/90 ms, flip angle = 90°, matrix size = 256 × 256, slice thickness = 4.0 mm, and *b* values of 0 and 850 s/mm^2^) collected before the contrast medium was injected. Part of the scanned image data is shown in Figure 1.

The article "Breast MRI Segmentation and Ki-67 High- and Low-Expression Prediction Algorithm Based on Deep Learning" was published in 2022. Journal: Comput Math Methods Med.

We defined three ROI regions (Figure 2). They are the tumor body, the stromal area around the tumor, and three ROIs that combine the two. The peritumor stroma was defined as a 5 mm expansion of the tumor boundary.

#### 2.1.2. Data Annotation

The tumor images we collected were manually delineated by two senior medical radiologists engaged in breast imaging diagnosis, and the molecular subtype labeling was based on the pathology report as the gold standard. In addition, corresponding contour labels are also made according to the boundaries of the tumor labels. The boundary of the contour label is represented by 1, and the area outside the boundary is represented by 0.

The scanned images often generate various noises due to external influences, so the images should be smoothed before training to remove the influential noises, so that the subsequent segmentation results are more accurate.

### 2.2. Improve Attention U-Net Network Model Implementation

U-Net is an upgraded network model based on FCN that comprises of a contraction (encoding) path and an expansion (decoding) path that are orthogonal to one another [34]. The shrinking path reduces the size of the input image by downsampling the feature map via consecutive convolutional layers and max-pooling layers; the expanding path restores the image size and information by upsampling the feature map through convolutional and deconvolutional layers. The encoder and decoder are connected by skip connection layer, and the image details lost during downsampling by the encoder are recovered. U-Net can achieve good performance when training samples with less data, so U-Net is widely used in medical-related fields. The U-Net structure is shown in Figure 3.

The human attention mechanism, which is commonly employed in deep learning, was used to name the attention model. In medical picture segmentation, an attention mechanism is included into the network structure to improve the model's sensitivity by highlighting the segmented object region and suppressing the feature response of irrelevant background regions. Inspired by attention U-Net [35], this paper improves on the original attention, and its structure is shown in Figure 4.

The article "Breast MRI Segmentation and Ki-67 High- and Low-Expression Prediction Algorithm Based on Deep Learning" was published in 2022. Journal: Comput Math Methods Med.

The attention mechanism takes two feature maps as input, one is the feature *x*_*l*_ in the skip connection, and the other is the feature *g*_*l*_ in the upsampling process; the input feature is linearly transformed by 1 × 1 convolution, and the size is unchanged, The feature maps whose number of channels is *C* are added together. Then, the intermediate feature map is obtained through the *SeLu* activation function, and after the 1 × 1 convolution operation, the Sigmoid function, and resampling, the graph attention coefficient ${\alpha_{l}}^{{}^{\circ}}{\hat{x}}_{l}$ is obtained as the output feature map, and its expression is

(1) $$\begin{array}{c} {\hat{x}}_{l}=\alpha_{l}∙x_{l}, \end{array}$$

where *x*_*l*_ is the input feature and *l* is the number of pixels in each feature.

The output result *x*_out_ of the attention mechanism is

(2) $$\begin{array}{c} x_{\text{out}}={\hat{x}}_{l}+g_{l}. \end{array}$$

In the segmentation task, due to the existence of multiple semantic categories, the coefficient of learning multidimensional attention is introduced, so the attention mechanism can pay more attention to the main situation in the segmentation process. Comparing the methods and performances of the multiplicative attention and additive attention algorithms, it can be found that the additive attention algorithm has higher precision and better segmentation effect. The attention coefficient *α*_*l*_ is

(3) $$\begin{array}{c} \alpha_{l}=\sigma_{2}\left(\varphi \left(\sigma_{1}\left(\omega_{x}x_{l}+\omega_{g}g_{l}+b_{g}\right)\right)+b_{\varphi }\right). \end{array}$$

In the formula, *ω*_*x*_ is the weight of the input *x*_*l*_, *ω*_*g*_ is the weight of the input *g*_*l*_, *φ* is the standard convolution function, *b*_*g*_ is the offset value of *g*_*l*_, and *b*_*φ*_ is the bias value of *φ*. The input features *x*_*l*_, *g*_*l*_ provide the attention mechanism with contextual information, which can determine which of the input features are related to breast tumors. *α*_*l*_ weights the low-level features, thereby increasing the correlation and suppressing irrelevant background information, so as not to affect the network judgment.

### 2.3. SVM Principle

Support vector machine (SVM) has obvious advantages in small sample statistics and has the ability to avoid structural risks. While pursuing roughly correct classification, it can avoid overfitting to a certain extent and has the best prediction ability [36]. Support vector machines are divided into linearly separable and nonlinearly separable. The basic principle is to map the sample training data in the low-dimensional space to the high-dimensional space, so that the sample training data is linearly separable, and then, the boundary is linearly divided by the Equations (3) and (4) defines the minimization function for finding the optimal hyperplane margin and its constraints.

(4) $$\begin{array}{c} \underset{w,b}{\min}\frac{1}{2}{\left\|\overset{⟶}{w}\right\|}^{2}\text{ subject to the constraints}, \end{array}$$

(5) $$\begin{array}{c} y_{i}\left(\overset{⟶}{w}∙\overset{⟶}{x_{i}}+b\right), \end{array}$$

where *w* is the normal, *b* is the threshold, and *x*_*i*_ is each sample instance.

The article "Breast MRI Segmentation and Ki-67 High- and Low-Expression Prediction Algorithm Based on Deep Learning" was published in 2022. Journal: Comput Math Methods Med.

In this work, the support vector machine's kernel function is a polynomial kernel function, which is defined as

(6) $$\begin{array}{c} K\left(x,x_{i}\right)={\left[\left(x∙x_{i}\right)+1\right]}^{d}, \end{array}$$

where *d* is the power of the polynomial kernel function; the larger the *d*, the more complex the algorithm and the longer the running time.

### 2.4. A Framework for Breast Tumor Segmentation and Prediction Based on Combinatorial Models

This paper proposes a tumor segmentation and prediction framework based on a combination of improved attention U-Net and SVM. The suggested framework, as illustrated in Figure 5, is divided into two stages: preprocessing, feature extraction, and training to improve attention U-Net and SVM and segmentation and creation of final Ki-67 prediction findings.

First, the enhanced attention U-Net and SVM are trained to learn the mapping from the grayscale picture domain to the tumor label domain. Then, the labeled segmentation output and labels of the improved attention U-Net are fed into the SVM classifier to obtain accurate Ki-67 predictions.

In the segmentation process, the target image changes greatly, which increases the difficulty of segmentation. In order to reduce the loss of adjacent feature information between different subregions, this paper uses the residual multiscale pooling layer to extract information of different scales. The pooling model fuses the features of the pooling kernel with 4 different scales, 2 × 2, 4 × 4, 8 × 8, and 16 × 16 from top to bottom, to extract global contextual feature information. The four layers of the pyramid output feature maps of different scales. In order to keep the global feature weight unchanged, a 1 × 1 convolution operation is connected behind the four different layers to reduce the number of channels of the output feature map. Then, using bilinear interpolation, upsample the low-level feature map to acquire features of the same size as the input pooling layer's original feature map and superimpose the obtained feature map with the original feature map to build a multichannel multiscale feature map for picture segmentation.

The article "Breast MRI Segmentation and Ki-67 High- and Low-Expression Prediction Algorithm Based on Deep Learning" was published in 2022. Journal: Comput Math Methods Med.

### 2.5. Model Design Details

The encoding and decoding part of the original U-shaped network is replaced with a recurrent residual atrous convolutional network. The problem of gradient disappearance caused by too deep network layers is solved by introducing identity mapping; the underlying feature information is repeatedly extracted and accumulated by using the cyclic structure; the receptive field is further expanded without loss of information through hole convolution, which improves the correlation between the layers of the network strengthens the global connection, but it also brings problems such as over-extraction of features and noise interference. To address these issues, a multiscale attention mechanism is added to the encoding and decoding skip connection, which increases the weight of tumor feature information and combines the feature semantic information of high and low layers, reduces the amount of network model parameters that must be calculated, and improves the light and dark contrast segmentation.

The encoder consists of 4 groups of downsampling layers and convolutional layers. The sampling layer is composed of 2 parallel channels. The convolutional layer adopts the cyclic residual hole convolution module to optimize the network structure and adds Dropblock to the convolutional block. Prevent overfitting problems. The decoder consists of 4 sets of upsampling layers, a convolutional layer of size 3 × 3 and a convolutional layer of the highest layer of 1 × 1, which is used to restore the feature size and output the segmentation result. The encoder and the decoder are connected by a skip layer with an attention mechanism. This module is used to fuse the imaging background and tumor proportions to reduce the influence of background chaos on tumor morphology. Low-level feature semantic information is usually less precise as time goes on, while high-level feature semantic information is more precise as time goes on. The context feature extraction module is a residual multiscale feature pooling layer that uses multiscale pooling to aggregate information from diverse locations and then extracts global context information.

## 3. Results

### 3.1. Segmentation Evaluation Metrics

Coefficient of Dice similarity (DSC) is an index that measures the rate at which manual and automatic segmentation are repeated. It is defined as follows:

(7) $$\begin{array}{c} \text{DSC}=\frac{2\text{TP}}{\text{FP}+2\text{TP}+\text{FN}}. \end{array}$$

Here, TP, FP, and FN are the number of tumor points detected as true positive, false positive, and false negative, respectively.

The article "Breast MRI Segmentation and Ki-67 High- and Low-Expression Prediction Algorithm Based on Deep Learning" was published in 2022. Journal: Comput Math Methods Med.

The fraction of correctly segmented tumor points in the segmentation result of tumor points is known as positive predictive value (PPV), which is defined as:

(8) $$\begin{array}{c} \text{PPV}=\frac{\text{TP}}{\text{TP}+\text{FP}}. \end{array}$$

Sensitivity is the proportion of correctly segmented tumor points to the true value of tumor points, which is defined as

(9) $$\begin{array}{c} \text{Sensitivity}=\frac{\text{TP}}{\text{TP}+\text{FN}}. \end{array}$$

### 3.2. Segmentation Results of the Combined Model

We train and segment the collected breast tumor photos to test the combined model's segmentation effect and then provide the experimental results. The result graph clearly shows the segmentation effect, demonstrating the efficiency of our strategy. The segmentation results of image slices of Ki-67 highly expressed breast cancer samples are shown in Figure 6.

At the same time, we randomly chose some samples from scan images of breast cancer with low Ki-67 expression for testing in order to confirm the efficiency of our procedure once more. The segmentation of image slices of breast cancer samples with low Ki-67 expression is shown in Figure 7.

It can be seen from the figure that our network can effectively segment breast tumors. Therefore, our network is very effective for the segmentation of breast tumors.

### 3.3. Comparison with Existing Methods

To demonstrate the usefulness of our suggested method, we compare it to methods proposed by other researchers, and the results of the comparison are shown in Table 1. Among them, Dalmış et al. [37] applied U-Net neural network. They segmented breast and FGT in MRI in datasets containing various MRI protocols and breast densities. Baccouche et al. [38] proposed an architecture called Connected-U-Nets, which uses other modified skip connections to connect two U-Nets. Haq et al. [39] proposed an automatic breast tumor segmentation segmentation method using conditional GAN (cGAN). It can be seen from the results in Table 1 that the combined framework proposed in this paper outperforms other methods in DSC, PPV, and sensitivity, which proves the feasibility of our method.

At the same time, in order to prove the universality of our combined network, we compare it with the traditional network. The experimental results are shown in Table 2. At the same time, in order to see the performance improvement of our combined network more intuitively, we calculated the improvement of the evaluation indicators, as shown in Table 3.

The article "Breast MRI Segmentation and Ki-67 High- and Low-Expression Prediction Algorithm Based on Deep Learning" was published in 2022. Journal: Comput Math Methods Med.

## 4. Discussion

Breast cancer is a very heterogeneous tumor with a wide range of morphologies, therapeutic responses, and patient outcomes due to distinct molecular subgroups. Ki-67 is a commonly used immunohistochemical marker in breast cancer detection, and its expression level is closely related to the invasiveness, type, treatment effect, and prognosis of breast cancer. However, in clinical practice, the expression of Ki-67 in the tumor can only be obtained through postoperative pathological tissue staining and immunohistochemical analysis and treatment are important. Magnetic resonance imaging (MRI) DWI can quantify the apparent diffusion coefficient (ADC) in the absence of a contrast agent, which reflects the movement of free water molecules in the tumor and provides information about tumor biology and microstructure. Texture analysis can capture microscopic features unrecognizable to the human eye in magnetic resonance imaging, quantifying tumor heterogeneity.

DWI can employ the diffusion motion of water molecules to display spatial information and cell density in human tissues at the molecular level, making it a useful MRI-assisted diagnostic procedure. In clinical practice, the most typically utilized ADC value is to quantify the diffusion degree of tissue water molecules. The ADC value of the Ki-67 high-expression group was lower than that of the low expression group ((0.820.08)10^−3^ vs. (0.980.15)10^−3^ mm^2^/s, *P* = 0.001), and the ADC value was inversely connected with Ki-67 expression (*r* = −0.514, *P* = 0.05), according to the findings. That is, the higher the Ki-67 index value, the lower the ADC value. At present, breast MRI scan and dynamic enhancement DWI scan are mostly used in clinical practice, which can obtain relatively complete imaging-related data of breast lesions, which further improves the diagnostic efficiency of breast cancer. It can distinguish between lesions and surrounding tissues and can also semiquantitatively or quantitatively evaluate the hemodynamic characteristics of breast lesions, which has high sensitivity for qualitative diagnosis of breast diseases.

Similar to other researchers, our method also suffers from certain limitations. The attention module used in this paper makes the segmentation model pay more attention to the local feature information of the tumor nucleus and the enhanced tumor region, ignoring the global feature information of the whole tumor, resulting in a slight decrease in the segmentation effect of the whole tumor. In the future segmentation model research, the local feature-level global feature information of tumor segmentation will be fused at the same time, in order to improve the segmentation accuracy of the whole tumor [40]. Note that volumetric modelling and visualization [41, 42] pertaining to the breast tumor structures can help in the analysis of breast cancer for future implementation. In addition, the consideration of harnessing the extreme learning methods [43] for segmentation used in this research may also be proposed as future work, and will enhance medical evaluation as well.

The article "Breast MRI Segmentation and Ki-67 High- and Low-Expression Prediction Algorithm Based on Deep Learning" was published in 2022. Journal: Comput Math Methods Med.

## 5. Conclusion

This paper proposes a tumor segmentation and prediction framework based on a combination of improved attention U-Net and SVM. This method outputs the segmentation results and labels of a learned improved attention U-Net into a SVM. During the training phase, we introduce coefficients for learning multidimensional attention. Focus on the main situation in the segmentation process through the attention mechanism. In order to achieve accurate prediction of Ki-67 high and low expression, we trained a support vector machine. The labeling output of the improved attention U-Net is sent to the SVM classifier for accurate classification. The method can adapt to the difference of breast tumors and segment breast tumors accurately and efficiently. In the follow-up research, we will explore attention U-Net in conjunction with other powerful classifiers. Compared with the segmentation frameworks of other papers, it is found that the DSC, PPV, and sensitivity of our combined model are 0.94, 0.93, and 0.94, respectively, with better segmentation performance and can generate accurate segmentation of breast tumors.

## Figures and Tables

**Figure 1:** Partially scanned image based on (a) Ki-67 highly expressed DWI sequence and (b) 2. Ki-67 low-expression DWI sequence.

**Figure 2:** Three ROI regions based on (a) tumor body, (b) the stromal area around the tumor, and (c) a combination of both.

**Figure 3:** CNN network structure diagram.

**Figure 4:** Improved attention mechanism.

**Figure 5:** A framework for breast tumor segmentation and prediction based on a combinatorial model.

**Figure 6:** Segmentation results of image slices of breast cancer samples with high Ki-67 expression based on (a) raw MRI scan image, (b) tumor segmentation results, (c) tumor boundary segmentation results, (d) tumor and boundary segmentation results, and (e) schematic overlay.

**Figure 7:** Segmentation results of image slices of breast cancer samples with low Ki-67 expression based on (a) raw MRI scan image, (b) tumor segmentation results, (c) tumor boundary segmentation results, (d) tumor and boundary segmentation results, and (e) schematic overlay.

**Table 1:** Comparison of different algorithms.

Method	Literature	DSC	PPV	Sensitivity
U-Net	Dalmış et al. [37]	0.87	0.86	0.89
Connected-U-Nets	Baccouche et al. [38]	0.89	0.90	0.91
BTS-GAN	Haq et al. [39]	0.90	0.92	0.91
CNN+SVM	Our method	0.94	0.93	0.94

The article "Breast MRI Segmentation and Ki-67 High- and Low-Expression Prediction Algorithm Based on Deep Learning" was published in 2022. Journal: Comput Math Methods Med.

**Table 2:** Compared with traditional network.

Method	DSC	PPV	Sensitivity
U-Net	0.80	0.81	0.80
V-Net	0.83	0.83	0.84
CNN	0.86	0.88	0.87
FCN	0.90	0.92	0.91
CNN+SVM	0.94	0.93	0.94

**Table 3:** Performance boost.

	U-Net	V-Net	CNN	FCN
DSC (↑)	0.14	0.11	0.08	0.04
PPV (↑)	0.12	0.10	0.05	0.01
Sensitivity (↑)	0.14	0.10	0.07	0.03

## Data Availability

Data available on request from the authors due to privacy/ethical restrictions.
